The article "“Bacterial Consortium”: A Potential Evolution of Fecal Microbiota Transplantation for the Treatment of Clostridioides difficile Infection" was published in 2022. Journal: Biomed Res Int.

# “Bacterial Consortium”: A Potential Evolution of Fecal Microbiota Transplantation for the Treatment of *Clostridioides difficile* Infection

**DOI:** 10.1155/2022/5787373

**Published:** 2022-08-08

**Authors:** Gianluca Quaranta, Gianluca Ianiro, Flavio De Maio, Alessandra Guarnaccia, Giovanni Fancello, Chiara Agrillo, Federica Iannarelli, Stefano Bibbo, Amedeo Amedei, Maurizio Sanguinetti, Giovanni Cammarota, Luca Masucci

**Affiliations:** ^1^Department of Laboratory and Infectious Sciences, A. Gemelli University Hospital IRCCS, 00168 Rome, Italy; ^2^Digestive Disease Center, A. Gemelli University Hospital IRCCS, Catholic University of Sacred Heart, 00168 Rome, Italy; ^3^Department of Experimental and Clinical Medicine, University of Florence and Department of Biomedicine, University Hospital Careggi (AOUC), 50139 Florence, Italy; ^4^Department of Basic Biotechnological Sciences, Intensivological and Perioperative Clinics, Catholic University of Sacred Heart, 00168 Rome, Italy

## Abstract

Fecal microbiota transplantation (FMT) consists of infusion of feces from a donor to a recipient patient in order to restore the resident microbial population. FMT has shown to be a valid clinical option for *Clostridioides difficile* infections (CDI). However, this approach shows several criticalities, such as the recruiting and screening of voluntary donors. Our aim was to evaluate the therapeutic efficacy of a synthetic bacterial suspension defined “Bacterial Consortium” (BC) infused in the colon of CDI patients. The suspension was composed by 13 microbial species isolated by culturomics protocols from healthy donors' feces. The efficacy of the treatment was assessed both clinically and by metagenomics typing. Fecal samples of the recipient patients were collected before and after infusion. DNA samples obtained from feces at different time points (preinfusion, 7, 15, 30, and 90 days after infusion) were analyzed by next-generation sequencing. Before infusion, patient 1 showed an intestinal microbiota dominated by the phylum *Bacteroidetes*. Seven days after the infusion, *Bacteroidetes* decreased, followed by an implementation of *Firmicutes* and *Verrucomicrobia*. Patient 2, before infusion, showed a strong abundance of *Proteobacteria* and a significant deficiency of *Bacteroidetes* and *Verrucomicrobia*. Seven days after infusion, *Proteobacteria* strongly decreased, while *Bacteroidetes* and *Verrucomicrobia* increased. Metagenomics data revealed an “awakening” by microbial species absent or low concentrated at time T0 and present after the infusion. In conclusion, the infusion of selected bacteria would act as a trigger factor for “bacterial repopulation” representing an innovative treatment in patients with *Clostridioides difficile* infections.

The article "“Bacterial Consortium”: A Potential Evolution of Fecal Microbiota Transplantation for the Treatment of Clostridioides difficile Infection" was published in 2022. Journal: Biomed Res Int.

## 1. Introduction

The human gut microbiota is composed by approximately 10^14^ commensal microorganisms including bacteria, viruses, fungi, and protozoa which represent a real solid organ, with an approximate weight of two kg [1]. Among these, bacteria represent the most studied group. The major representative phyla are *Firmicutes* and *Bacteroidetes* [2]. These microbial communities are highly organized and play a key role in modulating host immunity, nutrition, and metabolism and in the health/disease balance. Nowadays, it is well known that many intestinal and extraintestinal disorders are closely related to compositional and functional changes in commensal microbiota [3]. An example is represented by *Clostridioides difficile* infection (CDI). *Clostridioides difficile* (*C. difficile*) is a Gram-positive, sporogenous, motile, obligate anaerobic, and toxin-producing bacterium, originally identified in 1935 as a member of the microbial flora of infants. The strain was called *Bacillus difficile* for the difficulty of isolating and culturing [4]. CDI is a nosocomial infection mainly due to prolonged exposure to antibiotic therapies or prophylaxis during the hospitalization [5]. Currently, 7 cases are described per 10.000 patients admitted to European hospitals [6]. The statistics are also similar for the American hospitals, in which *C. difficile* is the main cause of nosocomial infection with 14.000 deaths/year [6, 7]. Currently, the therapeutic CDI approach is based on antibiotic therapy. The drugs of choice are metronidazole, vancomycin, and fidaxomicin [5, 8]. The great impact on public health and the appearance of resistant strains has forced the scientific community to find alternative therapeutic approaches, including the recent fecal microbiota transplantation (FMT). The FMT consists of the infusion of feces from a healthy donor to a recipient patient in order to treat specific diseases associated with alterations of the intestinal microbiota (dysbiosis) [8, 9]. FMT has shown interesting and promising results about the efficacy and management of the patients. But, concerning on procedural safety, potential pathogen transmission, and standardizing workflow, some key points have to be improved [10]. Recruiting of voluntary donors is a very critical aspect in FMT flowchart. In fact, donors' selection is a very hard and rigorous process. At first, each donor undergoes a general questionnaire to exclude intestinal and extraintestinal disorders. Subsequently, on donor stool and blood sample are performed cultural, molecular, and serologic analyses in order to avoid any possible transmission during infusion procedure [10–12]. It is clear that during screening process, a donor may result as unsuitable and, then, his fecal matter is unusable for the therapy. Based on current evidence, FMT represents an alternative safe therapeutic method with few adverse effects. Even so, every patient candidate for FMT needs to be informed about the potential risks before the procedure. Most clinical trials and systemic reviews presented that some minor adverse events, such as abdominal discomfort, diarrhea, constipation, and low-grade fever, were transiently noted after FMT, and uncommon severe side effects were often associated with the possible complications of endoscopy and sedation [13]. Moreover, some case reports describe a small population of patients that experienced IBD flares after FMT. The definite mechanism of IBD flare after FMT is still unclear, although Quera et al. suggested that transient bacteremia may result in altered intestinal permeability, resulting in a flare [14]. To date, long-term, follow-up studies (3–68 months post-FMT, average 17 months post-FMT) have found FMT to be relatively free of adverse effects [15]. The randomized control trial for treatment of rCDI (recurrent *Clostridioides difficile*) published by Van Nood et al. found that of the 16 patients treated, 15 experienced diarrhea, 5 had abdominal cramping, 3 had belching, and 1 had nausea. These effects were not observed in the control group that received only a bowel lavage; however, the effects were all self-limiting and resolved within 3 h post-FMT [16]. In terms of long-term adverse effects of FMT, there is a theoretical possibility that an infection will be transferred or a chronic disease will be stimulated (e.g., obesity, diabetes, and atherosclerosis) because of the alteration of the gut microbiota. However, long-term, follow-up studies are necessary to assess these risks. Advances in FMT delivery may reduce procedural complications in the future. Overcoming the possible occurrence of such adverse effects, in most cases mild and self-limiting, represents the main challenge for future FMT clinical applications. For these reasons, our study has been directed on the therapeutic efficacy of a synthetic bacterial preparation, called “Bacterial Consortium” (BC), in patients with CDI in substitution of the standard FMT. To this end, more than 60 different species of bacteria, both obligate and facultative anaerobes, normally present in the human intestinal microbiota, were isolated from healthy donors' stool samples (Figure 1). This stool substitute preparation is composed by 13 gut bacteria isolated in pure culture (Table I) from three healthy donors using culturomics' approach. Bacteroides strains were tested for susceptibility and resistance profile to antibiotics based on EUCAST guidelines. Culturomics is a set of culture conditions applied to isolate bacterial strains considered uncultivable [17]. Culture conditions include broth media enrichment, blood cultures' bottle, and selective and nonselective agar media incubated at different temperatures and times and observed from few days to months. Each colony is then identified by MALDI-TOF mass spectrometry [18–20]. Here, we reported the successful outcome of two patients with recurrent CDI unresponsive to conventional therapy and treated with BC infusion. Moreover, we provided the characterization by metagenomics of the recipient gut microbiota at different time points: preinfusion (T0), 7, 14, 30, and 90 days after transplantation (T1, T2, T3, and T4) in order to evaluate the following: (a) the engraftment of the infused bacterial species and (b) the richness and biodiversity of the bacterial communities pre- and post-FMT.

The article "“Bacterial Consortium”: A Potential Evolution of Fecal Microbiota Transplantation for the Treatment of Clostridioides difficile Infection" was published in 2022. Journal: Biomed Res Int.

## 2. Materials and Methods

### 2.1. Donors' Recruitment

Three donors (a 45-year-old woman, a 42-year-old woman, and a 43-year-old man) were recruited basing on their medical and clinical history at CEMAD Department in A. Gemelli Hospital (Rome) (protocol code 0021125/16) [8]. The relative fecal samples were analyzed in order to exclude the presence of *C. difficile* toxin A/B producer (Liaison, DiaSorin Spa, Saluggia VC, Italy) and intestinal pathogens such as *Salmonella* spp., *Campylobacter* spp., *Shigella* spp., *Yersinia enterocolitica*, protozoa, and helminths. The presence of vancomycin-resistant Enterococci (VRE), methicillin-resistant Staphylococcus aureus (MRSA), and Gram-negative multi-drug-resistant bacteria (MDR) was also excluded by cultural assay. Moreover, RT-PCR Allplex™ Gastrointestinal Panel Assays (Seegene, South Korea) for the comprehensive detection and identification of 25 gastrointestinal pathogens (virus, bacteria, toxins and parasite) were performed in order to declare the stool “pathogens free” and then suitable for infusion.

### 2.2. Culturomics Protocol

Thirty grams of fecal sample was suspended in 30 mL of saline solution. After the homogenization by Stomacher® 400 Circulator (SEWARD, UK), the fecal suspension was split in two aliquots and centrifuged at 3500 × g for 10 minutes [21]. Supernatants were discarded, and the two pellets were resuspended: one in 15 mL of rumen fluid and the other one in 15 mL of supplemented Brucella Broth (BB, Remel INC., Lenexa, USA). Each enriched suspension (5 mL) was divided into six 2.5 mL aliquots, which were inoculated into a bottle of blood cultures for aerobes and anaerobes (Becton, Dickinson and Company, Benex Limited, Shannon, Ireland). Subsequently, the bottles were incubated at 30°C, 37°C, and 42°C for seven and fourteen days. After incubation period, 10 *μ*L of bacterial enriched suspension was plated on the following agar media and then incubated: TSA (Tryptic Soy Agar, Becton Dickinson, Franklin Lakes, USA), SCH (Schaedler agar, Becton Dickinson, Franklin Lakes, USA), CNA (Columbia agar, Becton Dickinson, Franklin Lakes, USA), and PVX (chocolate agar, bioMérieux, Marcy-l'Étoile, France). Culture conditions are described in Figure 2.

The article "“Bacterial Consortium”: A Potential Evolution of Fecal Microbiota Transplantation for the Treatment of Clostridioides difficile Infection" was published in 2022. Journal: Biomed Res Int.

### 2.3. Identification of Isolated Strains

Each colony observed after the incubation phase was first isolated in order to obtain a pure culture and subsequently identified by MALDI-TOF mass spectrometry (Bruker Daltonics, Billerica, MA, USA). The bacterial colonies were “spotted” on the target plate and hydrated with 1 *μ*L of *α*-cyrano-4-hydroxycinnamic acid (*α*-CHCA). Before each measurement, the instrument was calibrated using Bacterial Test Standard (BTS, Bruker Daltonics, Billerica, MA, USA). All the bacterial strains analyzed reported an identification reliability score greater than 1.9. Bacterial strains of interest were stored at -80° C and in 10% glycerol suspension. Antibiotic susceptibility tests were performed on the thirteen strains selected in order to avoid the infusion, in the recipient patient, of any MDR microorganisms. MICs were obtained by broth microdilution method (Sensititre™ Anaerobe MIC Plate, Thermo Fisher Scientific, Waltham, Massachusetts, USA) and epsilon test (E-test, bioMerieux, Marcy-l'Étoile, France) (data not shown).

### 2.4. “Bacterial Consortium” Preparation

The preparation of the synthetic suspension was carried out on the same day on which the infusion was scheduled. The thirteen selected species were cultured under anaerobic conditions 72 h before infusion in order to obtain bacterial suspensions (16 mL of 0.9% saline solution) prepared considering turbidity values (McFarland) between 2.5 and 5 McFarland equal to about 5 × 10^8^-10^9^ CFU/mL. The thirteen suspensions were combined in a single solution with a final volume of 250 mL. The preparation was poured into a sterile glass bottle and incubated for 30 minutes at 37°C.

### 2.5. Infusion Procedure

The recipient patients (PZ1 = female 80 years; PZ2 = female 70 years) underwent pretreatment with vancomycin (125 mg orally, 4 times/day for 3 days) followed by intestinal washing, on the last day of antibiotic therapy, with Macrogol (SELG ESSE). On day 4, the bacterial suspension synthesized in the laboratory was infused about an hour before surgery. The solution was infused, using 50 mL syringes, at the level of the proximal section of the colon. During the operation, the patient was placed on his right side. The same position was maintained for at least 1 h postsurgery in order to implement the permanence of the infused material in the colon. The whole procedure lasted about 10 minutes. At the end of the entire procedure, the patient was monitored for two hours [5, 8].

The article "“Bacterial Consortium”: A Potential Evolution of Fecal Microbiota Transplantation for the Treatment of Clostridioides difficile Infection" was published in 2022. Journal: Biomed Res Int.

### 2.6. DNA Extraction and Metagenomics Analysis

Metagenomics evaluation was carried out on fecal samples from two recipient patients and collected at different time points: pretransplantation (T0), 7 days (T1), 15 days (T2), 1 month (T3), and 3 months (T4) posttransplantation. Acid nucleic extraction from stool samples was performed using DANAGENE Microbiome Fecal DNA Kit (Danagen, Barcelona, Spain). Briefly, 50-200 mg of fecal matter was weighed and placed into a bead microtube in order to ensure cell lysis. Subsequently, 25 *μ*L of proteinase K was added to the lysate to remove RNase and DNase activities. A washing phase was performed using a DNA column-collection tube. Lastly, 200 *μ*L of Elution Buffer was added in order to obtain the same volume of purified DNA. DNA samples were analyzed using the KIT 16S rRNA MiSeq (Illumina). The amplified target regions correspond to the variable regions V3-V4. In a first phase, the DNA was amplified using two specific primers for the V3-V4 regions, which have structures defined as adapters (forward primer 5′TCGTCGGAGCAGCTGTGTGTATAAGAACACCTGGGNCAG; reverse 5′TCGTCGGCAGCGCTCGGAGATGTTTAGAGAGAGACGACT). Each reaction had a final volume of 25 *μ*L of which are 12.5 *μ*L of 2X Kapa HiFi HotStart mix (Anachem, Dublin, Ireland), 5 *μ*L primer F (1 *μ*M), 5 *μ*L primer R (1 *μ*M), and 2.5 *μ*L of DNA. The amplification reaction was carried out with the following thermal profile: heated lid 110°C, 95°C × 3 min, 95°C 30 sec, 55°C × 30 sec, and 72° × 30 sec for 25 cycles followed by a final extension phase at 72°C × 5 min. The PCR products were visualized by agarose gel electrophoresis (1X TAE, 1.5% agarose, 90 V) and subsequently purified by AMPure XP bead purification (Labplan, Dublin, Ireland). A second PCR was conducted on the purified DNA. Each reaction involved the use of 5 *μ*L of primer index 1 (N7xx), 5 *μ*L of primer index 2 (S5xx), 25 *μ*L of 2X Kapa HiFi, and 10 *μ*L of water. The PCR products were visualized by agarose gel electrophoresis as previously described. The samples were quantified by Qubit (Bio-Sciences, Dublin, Ireland) and then collected in equimolar concentration. The sample pool (4 nM) was denatured using 0.2 N NaOH and subsequently diluted to 4pM and combined with PhiX 4p M. The samples were sequential via the MiSeq platform using 2 × 300 V3 kit cycles following the standard Illumina protocol [22–24].

The article "“Bacterial Consortium”: A Potential Evolution of Fecal Microbiota Transplantation for the Treatment of Clostridioides difficile Infection" was published in 2022. Journal: Biomed Res Int.

### 2.7. Bioinformatics Analyses

Raw sequencing data were demultiplexed and FastQ were analyzed by using Qiime2 pipeline. Briefly, FastQ reads were trimmed to remove Illumina adapters and nonbiological primer sequences and then quality filtered. Amplicon Sequence Variants (ASVs) and chimera removing were performed by DADA2 algorithm. Taxonomic annotation was obtained by using VSearch and SILVA 132 database. Final data were preprocessed removing mitochondrial sequences and taxa represented under 0.01%. Statistical analysis of microbiota diversity was performed in R studio (https://www.rstudio.com/; version 4.0.2) using phyloseq package. Alpha diversity was evaluated by observed richness, Shannon index, and Pielou's evenness on rarefied data. Statistical significance for each time point of the single patient was assessed by Kolmogorov-Smirnov tests, assuming significant results with a *p* < 0.05.

## 3. Results

### 3.1. Culturomics

Through “culturomics,” 60 bacterial species (data not shown) from the stool of the healthy donors have been isolated and collected. Among these, 13 bacterial strains (Table 1) with different microbial properties were selected in order to create a bacterial solution to be infused in CDI patients. Antibiotic susceptibility tests were performed by triplicate E-test on Bacteroides strains and valuated by EUCAST guidelines.

### 3.2. Clinical Outcome

The patients were monitored two hours following the infusion, and no adverse events were noted. Subsequently, patients were evaluated one week after procedure by anamnestic visit in which no complications such as diarrheal discharge, fever, or abdominal pain were reported. The clinical evaluation was carried out up to three months after the infusion giving positive results.

### 3.3. Phylum Modulation

Figure 3 shows the time-course modulation of the phyla in PZ 1. Before FMT (T0), its gut microbiota was mainly characterized *Bacteroidetes* (72%). *Firmicutes* and *Proteobacteria* were present with a relative abundance of 12% and 10%, respectively. *Verrucomicrobia* at T0 were present in percentages close to zero (0.01%). At T1 (7 days), there is a series of changes in the PZ1 microbiota. Specifically, *Bacteroidetes* underwent a decrease of 25% reaching 47% followed by an increase of *Firmicutes* (23%) and *Verrucomicrobia* (from 0.01% to 22%). In the subsequent time points, there appeared a stabilization of the intestinal populations in which *Bacteroidetes* and *Firmicutes* (63% and 33%) increased and the *Proteobacteria* reached minimum values (from 10% at T0 to 4% at T4).

The article "“Bacterial Consortium”: A Potential Evolution of Fecal Microbiota Transplantation for the Treatment of Clostridioides difficile Infection" was published in 2022. Journal: Biomed Res Int.

Regarding the FMT, PZ 2 showed a gut microbial pattern characterized by a strong abundance of *Proteobacteria* (60%) and *Firmicutes* (40%) and a significant deficiency of *Bacteroidetes* (0.05%) and *Verrucomicrobia* (0.02%). After seven days, *Proteobacteria* underwent a decline from 60% to 5%, while *Bacteroidetes* increased to almost 50% of the relative abundance accompanied by an implementation of *Verrucomicrobia* (17%). Three months after infusion, microbiota appeared stabilized with a prevalence of *Bacteroidetes* and *Firmicutes* (50% and 46%).

### 3.4. Richness and Biodiversity

Figure 4 shows the number and the distribution of microbial species detected in the samples of the two patients at the different time points. At T0, PZ 1 (sample 1) and PZ 2 (sample 2) were characterized by 27 and 46 species, respectively. In the subsequent time points, biodiversity increased passing up to 70 species detected at T4 for both patients (Figure 4(a)). Moreover, diversity along species was evaluated with Shannon and evenness index (Figures 4(b) and 4(c)). Finally, Figure 5 describes the relative abundance of beneficial bacteria such as *Akkermansia muciniphila*. This bacterium was absent at T0 in both patients. After infusion (in detail at T1), *Akkermansia muciniphila* raised concentrations of 22% in patient 1 and 17.5% in patient 2.

## 4. Discussion

The *Clostridioides difficile* infection is a nosocomial infection due to prolonged exposure to antibiotics [25, 26]. In the last decade, the CDI is involving also younger people not undergoing antibiotic therapies [7]. The clinical severity ranges from mild to severe diarrhea up to leading to toxic megacolon and intestinal perforation [27–30].The pathogenesis of CDI depends not only on toxins production but also on the intestinal microenvironment. In fact, recently, several studies have shown how different metabolites and several groups of microorganisms may contribute to the inflammatory state described in CDI [31].

Specifically, it has been shown that *C. difficile* spores' germination is sensitive to the presence of primary bile acids such as cholate and taurocholate produced by the liver and secondary bile acids such as deoxycholate. In fact, these molecules are abundant in healthy subjects compared to subjects with recurrent infection. On the other hand, the inflammatory state of CDI and other inflammatory bowel disorders such as UC and IBD is triggered by the activity and overgrowth of certain microbial groups. It is evident how sulfate-reducing bacteria (SRB), a small group of anaerobic bacteria including *Desulfovibrio desulfuricans*, appear overexpressed in patients with inflammatory syndromes. These bacteria, being resistant to broad-spectrum antibiotics, may overgrow in patients treated with antibiotic therapy, contributing to intestinal inflammation through the production of high levels of H_2_S or through their cytotoxic activity against epithelial cells [32, 33]. In this scenario, FMT is thriving as a valid therapeutic approach to CDI with an 80% efficacy when antibiotic therapies fail [5]. The preparation of fresh or frozen fecal suspensions requires the constant and periodic presence of donors. In addition, these donors must result negative for a series of serological and microbiological screening tests [8]. Moreover, stool sample must be processed within six hours after defecation in order to preserve anaerobes [8, 10]. All these aspects make the procedure laborious and poorly standardized. Furthermore, it is essential to know in detail the bacterial composition of the suspension to be infused into the recipient in order to increase the efficacy and especially the safety of the treatment. All these mentioned technical, logistical, and bureaucratic criticalities mean that not all healthcare facilities can offer their patients this important therapeutic option. In this study, our aim was to develop a “home-made” bacterial suspension, defined “Bacterial Consortium,” bypassing all the lacks of classical FMT procedure. In 2013, Petrof et al. have worked on formulating a synthetic ecosystem called RePOOPulate, consisting of a series of bacterial strains previously tested for antibiotic resistance [34]. This preparation was infused by colonoscopy in two patients affected by recurrent CDI with the clinical resolution in both cases [35].

The article "“Bacterial Consortium”: A Potential Evolution of Fecal Microbiota Transplantation for the Treatment of Clostridioides difficile Infection" was published in 2022. Journal: Biomed Res Int.

In our work, the first step was the selection of “beneficial bacteria” from the gut of healthy donors. Culturomics was the main strategy to isolate and collect bacterial strains. Of course, this method is very laborious and provides long time to result. But, on the other hand, a very interesting strategy is to describe microbial populations in a specific body district [17, 34]. In fact, thanks to a variety of enrichment factors and growth conditions, it is possible detecting microbial species present in low concentrations [17]. A profoundly different approach is metagenomics. This method is characterized by many strengths and weaknesses. Specifically, metagenomics allows the inclusion of a large number of sample and a “relative” rapid analysis in comparison to culturomics. But, the most crucial weaknesses are represented by (i) the depth limit in detection, (ii) minority populations are insufficiently detected, and (iii) the impossibility to discriminate between live bacteria and transient DNA [36]. This pilot study shows that a “synthetic” suspension may be a valid alternative option to the use of feces from a healthy donor. Considering the definition of recurrent CDI as an infection that recurs within 8 weeks after the onset of a previous episode, both patients were monitored up to three months after the procedure. They did not show diarrhea episodes, gastrointestinal symptoms, and positive laboratory tests during the entire follow up (7, 15, 30, and 90 days). In addition, metagenomics analysis showed a marked gut microbiota shaping after infusion. Specifically, a resettlement of the microbial populations was observed in both patients as demonstrated by the negative result for *C. difficile* toxin detection and by an increased number of detected bacterial species. Among these species appeared both the strains infused with BC and other species, absent or low concentrated before infusion, such as *Akkermansia muciniphila*. This bacterium stimulates communication between the bacteria in the intestinal microbiota and improves the function of the gut barrier by enhancing immune response. In addition, it is able to influence the metabolism of sugars and fats generating molecules acting as postbiotics [37]. Moreover, in both patients, the percentage of the phylum Proteobacteria appears dramatically reduced after infusion. The Proteobacteria group is mainly represented by Gram negative bacteria which contribute to the typical CDI inflammatory status [38]. The increase of species reported in Figure 3 is an evidence of a “microbial awakening” in which gut microbiota reverts to eubiosis conditions with an increment of the percentage of *Firmicutes* and *Bacteroidetes*. These data suggest a modulatory and stimulatory action of the “Bacterial Consortium” on the resident microbiota damaged by the pathological action of *C. difficile*. The use of a synthetic preparation, composed exclusively of bacteria, reveals numerous potential advantages. First of all, knowing the real composition of the infused suspension offers more control over procedure and consequently a wider safety standard compared to the infusion of fecal matter. Furthermore, knowing the bacterial components infused ensures a high degree of methodological reproducibility. The efficiency of the classic FMT is strongly influenced by the sampling and delivery phase of the feces in the laboratory. Using cultivable bacteria could allow to bypass this logistic problem and to have stable bacterial strains whenever necessary.

The article "“Bacterial Consortium”: A Potential Evolution of Fecal Microbiota Transplantation for the Treatment of Clostridioides difficile Infection" was published in 2022. Journal: Biomed Res Int.

## 5. Conclusion

This study shows some limits, especially the restricted number of recruited patients, but the principal aim of this explorative pilot study was the development of efficacious alternative to FMT. Our future proposal will be enrolling more patients in order to extend this therapeutic option not only to CDI but also for other gastrointestinal disorders. In the personalized medicine era, “Bacterial Consortium,” supported by culturomics and metagenomics, could be a revolutionary choice to treat patients with intestinal dysbiosis and hopefully extraintestinal disorders.

## Figures and Tables

**Figure 1:** Study design. Candidate donor undergoes multistep screening to exclude risk factors, comorbidities, and any potential pathogen transmission. Subsequently, feces from a “healthy donor” are processed for culturomics in order to collect potential beneficial bacteria.

**Figure 2:** Culturomics protocol conditions used for bacterial isolation and BC synthesis.

**Figure 3:** Relative abundance at phylum level in PZ 1 (sample 1) and PZ 2 (sample2).

**Figure 4:** Alpha diversity analysis of fecal bacterial communities after fecal microbiota transplantation. Species richness (a), Shannon diversity index (b), and equitability, as Pielou's evenness values (c) were compared among T0 (before fecal transplantation) and T1-3 (after fecal microbiota transplantation).

**Figure 5:** Relative abundance of *Akkermansia muciniphila* in PZ1 (sample 1) and PZ 2 (sample 2).

**Table 1:** List of bacterial strains isolated by culturomics and relative concentrations in BC and MIC values obtained by Epsilon tests performed in triplicate. MER: meropenem; CLI: clindamycin; MRD: metronidazole; TZP: piperacillin-tazobactam; not applicable: there are no EUCAST clinical breakpoints for these strains.

Bacterial strain	Concentration (CFU/mL)	MIC values
*Acidaminococcus intestini*	5 × 10^8^	Not applicable
*Bacteroides fragilis*	5 × 10^8^	MER 1 S CLI 64 R MRD 1 S TZP 4 S
*Bacteroides ovatus*	5 × 10^8^	MER 0.25 S CLI 4 S MRD 8 R TZP 4 S
*Bacteroides uniformis*	5 × 10^8^	MER 0.25 S CLI 2 S MRD 4 S TZP 4 S
*Bifidobacterium longum*	5 × 10^8^	Not applicable
*Clostridium scindens*	5 × 10^8^	Not applicable
*Lactobacillus casei*	5 × 10^8^	Not applicable
*Lactobacillus gasseri*	5 × 10^8^	Not applicable
*Lactobacillus rhamnosus*	5 × 10^8^	Not applicable
*Lactobacillus parabuchneri*	5 × 10^8^	Not applicable
*Parabacteroides distasonis*	5 × 10^8^	Not applicable
*Propionibacterium avidum*	5 × 10^8^	Not applicable
*Ruminococcus gnavus*	5 × 10^8^	Not applicable

## Data Availability

The datasets used and/or analyzed during the present study are available from the corresponding author on reasonable request.
